# Active Management of Labor Process under Smart Medical Model Improves Vaginal Delivery Outcomes of Pregnant Women with Preeclampsia

**DOI:** 10.1155/2022/8926335

**Published:** 2022-04-07

**Authors:** Siming Xin, Xianxian Liu, Jiusheng Zheng, Hua Lai, Jiao Zhou, Feng Zhang, Xiaoying Wu, Ting Shen, Lin Xu, Xiaoming Zeng

**Affiliations:** ^1^Department of Obstetrics, Jiangxi Provincial Maternal and Child Health Hospital, Nanchang, China; ^2^Key Laboratory of Women's Reproductive Health of Jiangxi Province, Jiangxi Provincial Maternal and Child Health Hospital, Nanchang, China; ^3^Department of Science and Education, Jiangxi Provincial Maternal and Child Health Hospital, Nanchang, China

## Abstract

**Background:**

In a global environment of increasing cesarean delivery rate, promoting vaginal delivery, reducing the rate of first cesarean section, and the incidence of vaginal delivery complications are the objectives of obstetric medical quality and safety in China. As a common obstetric complication, preeclampsia affects the safety of many pregnant women. It is the obstetrician's great responsibility to promote vaginal delivery and improve delivery outcomes in preeclampsia. To this end, we explored the roles of active labor management under the smart medical model in improving the outcomes of vaginal delivery for pregnant women with preeclampsia.

**Methods:**

The clinical data of 219 cases of preeclampsia pregnant women who delivered vaginally in our hospital from January 2017 to December 2020 were retrospectively analyzed. According to different labor process management, they were divided into study group (active labor process management group) and control group (normal labor process management group). Active labor process management methods included intrapartum ultrasound, central fetal heart rate monitoring, Doula delivery, labor analgesia, and quality of life care. The differences in delivery process, delivery outcome, bleeding causes, and hemostatic measures were compared between the two groups.

**Results:**

(1) The incidence of preeclampsia in our hospital showed an increasing trend in recent four years; (2) in smart hospitals, the active management of labor process reduced the probability of transferring to the cesarean section in preeclampsia pregnant women with vaginal trial failure; and (3) active labor process management reduced the rate of lateral episiotomy, decreased the postpartum hemorrhage volume within two hours, and improved the vaginal delivery outcome of preeclampsia pregnant women.

**Conclusions:**

In the era of the rapid development of the Internet, vigorously promoting the construction of smart hospitals and actively managing the delivery process can reduce the failure rate of vaginal trial delivery and improve the outcomes of vaginal delivery in preeclampsia women.

## 1. Introduction

In recent years, with the rapid development of Internet technology, emerging technologies such as artificial intelligence, informatization, big data, and cloud computing have emerged, driving technological changes in the medical field. Smart medicine is an innovative application of the Internet in the medical field. Based on Internet technology, it deeply integrates with traditional medical services through information means, effectively connects patients, medical staff, medical equipment, and medical institutions, and realizes efficient coordination among various departments and personnel. This not only promotes the sharing and exchange of medical information and resources and improves the utilization rate of medical resources but also meets the needs of disease diagnosis and treatment of patients and improves their medical satisfaction. At present, smart medical research mainly covers electronic medical records, medical and health big data analysis and mining, intelligent medical image analysis, intelligent assisted diagnosis, intelligent diagnosis and treatment, etc. In obstetrics, the smart medical treatment has penetrated the prediction of preeclampsia [1, 2], placenta implantation [3], type of labor [4], fetal growth [5], and other aspects. At the same time, it also made some beneficial explorations in forceps delivery [6] and treatment of obstetric complications [7, 8].

Preeclampsia is a common obstetric complication with a global prevalence of 2%–8% [9, 10]. In China, with the liberalization of fertility policy and the development of assisted reproductive technology, the number of pregnant women of advanced age, assisted reproduction, multiple pregnancies, and overweight have increased significantly, and the incidence of preeclampsia is about 2.7% [11], which is one of the major causes of maternal and perinatal death [12]. At present, the common treatment regimen for preeclampsia is symptomatic treatment with sedation, antispasmodic, antihypertensive, and correction of hypoproteinemia, and the only effective intervention plan is the termination of pregnancy. The 2020 edition of the Chinese Medical Association's guidelines for the management of hypertensive disorders in pregnancy states that, in principle, vaginal delivery should be considered for pregnant women with preeclampsia who are not severely ill and who do not have an indication for cesarean delivery. However, in actual clinical practice, many pregnant women with preeclampsia who are eligible for vaginal trial of labor directly opt for cesarean section, or because of the imperfection of medical information systems and inadequate maternal-fetal monitoring, patients with preeclampsia undergo unnecessary conversion to cesarean section during the vaginal trial of labor. This has undoubtedly increased the cesarean section rate and the incidence of surgery-related complications in our country, aggravating the economic burden on maternal families and the country.

To effectively promote vaginal delivery and reduce the rate of first cesarean section and complications of vaginal delivery, our hospital launched the construction of smart hospital in 2018 and successively introduced the integrated platform, hospital information system, laboratory information management system, hospital resource planning, remote fetal heart rate monitor, and central fetal heart rate monitor. At the same time, we established a sound medical information system and fetal monitoring system. Since 2019, relying on the above intelligent systems and equipment, our hospital started to explore the active labor process management methods under the new labor guidelines for preeclampsia pregnant women. In this study, we retrospectively analyzed the clinical data of pregnant women with preeclampsia who delivered vaginally in our hospital from January 1, 2017, to December 31, 2020, to explore the effectiveness of active labor management in improving the delivery outcomes of pregnant women with preeclampsia.

## 2. Materials and Methods

### 2.1. Materials

This is a single-center retrospective case-control study. All medical records came from Jiangxi Provincial Maternal and Child Health Hospital and were retrieved through the electronic medical record system of the hospital. The retrieval strategies were as follows: preeclampsia as the discharge diagnosis, vaginal delivery as the delivery mode, and January 1, 2017, to December 31, 2020, as the delivery time. Inclusion criteria were as follows: singleton live birth, full-term pregnancy, and spontaneous delivery. Exclusion criteria were as follows: scarred uterus, poorly controlled blood pressure, severe impairment of organ function, chronic hypertension complicated with preeclampsia, and renal hypertension complicated with antiphospholipid antibody syndrome. A total of 219 pregnant women were enrolled in this study.

### 2.2. Diagnostic Criteria of Preeclampsia

The diagnosis of preeclampsia refers to the Guidelines for the Diagnosis and Treatment of Hypertensive Disorders in Pregnancy (2015) formulated by the Hypertensive Diseases Group in Pregnancy of the Chinese Society of Obstetrics and Gynecology. Systolic blood pressure ≥ 140 mmHg or diastolic blood pressure ≥ 90 mmHg at or after 20 weeks of pregnancy, together with one or more of the following new-onset conditions; urinary protein ≥ 3.0 g per 24 hours, urinary protein/creatinine ratio ≥ 0.3, random urinary protein ≥ (+) if quantitative urine protein detection is not available; no proteinuria but with damage to vital organs such as the heart, lung, liver, kidney, or involvement of the hematological system, nervous system, digestive system, and fetus, etc.

### 2.3. Definition of Each Stage of Labor

(1) The first stage of labor was known as the cervical dilation period, which referred to the process from regular uterine contractions to the full dilation of the cervix; (2) the second stage of labor was also known as the fetal delivery period, referred to the process from the full dilation of the cervix to the delivery of the fetus; and (3) the third stage of labor also known as the placental delivery period referred to the process from the delivery of the fetus to the delivery of the placenta.

### 2.4. Key Points of Labor Management in the Control Group

The treatment of labor process was performed according to the “Expert Consensus on New Labor Process Standards and Treatment (2014)” issued by the Obstetrics and Gynecology Group of the Chinese Medical Association's Obstetrics and Gynecology Branch. The main details were as follows:

1. Key Points of the First Stage of Labor Management. Vaginal palpation was used to assess the progress of labor, which included fetal position, fetal head position, and fetal lie. The criteria for abnormal labor were as follows: cessation of uterine orifice dilation, cessation of fetal head descent, and non-parallelism between fetal head height and uterine orifice dilation. The standard of parallelism between the height of fetal head and the dilation of the uterus is as follows, when uterine orifice dilation size was <3 cm, 3–4 cm, 5–6 cm, 7–8 cm, and 9–10 cm, and the corresponding fetal head position was S—3∼S—2, S—2∼S—1, S 0∼*S* + 1, *S* + 1 ∼ *S* + 2, and *S* + 2∼*S* + 3. The fetal heart rate monitoring was performed every 2 hours for duration of 20–40 minutes. The observation of labor progress and fetal heart rate was carried out by the resident physician in the delivery room. If there was any abnormality during labor, the attending physician with more than 5 years of delivery room work experience must check it again. When the final judgment was abnormal labor, interventions such as sedation, manual rupture of membranes, oxytocin drip, and transfer to cesarean section were taken according to the situation.
2. Key Points of the Second Stage of Labor Management. A bedside fetal monitor was used for continuous fetal heart rate monitoring. Doctors and midwives in the delivery room checked the fetal heart rate pattern timely to detect abnormalities as soon as possible and then actively adopt forceps or cesarean section to terminate pregnancy according to the situation.
3. Key Points of the Third Stage of Labor Management. When the fetal shoulder was delivered, 10–20 U oxytocin was used immediately. If necessary, 100 *μ*g carbetocin was injected intravenously after fetal delivery. If there was still active bleeding, 250 *μ*g carboprost trometamol was added. Excluding laceration of birth canal and residual placenta, if uterine bleeding persisted after the use of a variety of uterine contraction drugs and uterine massage to promote uterine contraction, uterine tamponade hemostatic treatments would be used as soon as possible.

### 2.5. Key Points of Labor Management in the Study Group

During the whole labor process, all patients were provided with professional, comprehensive, and humanized Doula delivery services by systematically trained Doula personnel to give patients physical, psychological, and emotional support. The main details of labor management according to the active labor management methods under the new labor standard were as follows:

1. Key Points of the First Stage of Labor Management. Under the premise of informed consent of patients, all pregnant women with preeclampsia were provided with intraspinal labor analgesia by an anesthesiologist in the delivery room. At the same time, life care would be strengthened, and feeding, fluid rehydration, and rest were encouraged during labor. The progress of labor was assessed by intravaginal palpation and ultrasound during labor. The model of the ultrasonic diagnostic apparatus was S8Exp, and the probe frequency was set as 2–4 mega-hertz. Transabdominal ultrasound was used to determine fetal position, and transperineal ultrasound was used to evaluate fetal head position. In transperineal ultrasound, the symphysis pubis and fetal head position of pregnant women were often used as markers. The content of the intrapartum ultrasound measurement included fetal head progression angle, midline angle, distance between fetal head and pubic symphysis, fetal head direction, and distance between fetal head and perineum. The fetal heart rate monitoring was performed by central fetal heart rate monitor, and the related parameters of fetal heart rate monitoring were the same as those of the control group. If there was any abnormality during labor, the resident physician would immediately contact the attending obstetrician who has been trained in systematic ultrasound to check again. If an abnormal labor did occur, interventions such as sedation, artificial rupture of membranes, oxytocin drip, and transfer to cesarean section were taken according to the situation.
2. Key Points of the Second Stage of Labor Management. The central fetal heart rate monitor was used to monitor the fetal heart rate continuously throughout the whole process. Once abnormal fetal heart rate monitor pattern occurred, the central monitor would open an alarm to remind the medical staff to take active measures.
3. Key Points of the Third Stage of Labor Management. The treatments were basically the same as the control group, except that delayed umbilical cord amputation and controlled cord pulling were encouraged when the mother and newborn were in stable condition.

### 2.6. Blood Pressure Management during Labor

For patients without organ dysfunction, the target blood pressure control value was 130–155/80–105 mmHg, and for those with organ dysfunction, the blood pressure control target value was 130–139/80–89 mmHg. During the first stage of labor, blood pressure was monitored every 2 hours to ensure the patient's rest and proper activities. During the second stage of labor, blood pressure was continuously monitored, and blood pressure was monitored every half hour during the third stage of labor. Of course, if blood pressure exceeded the target value during the monitoring period, the monitoring interval needed to be shortened accordingly.

### 2.7. Observed Indicators

Duration of 3 stages of labor, rate of forceps assisted delivery, rate of perineal laceration, rate of cervical laceration and placental abruption, postpartum hemorrhage volume within two hours, birth weight of the newborn, and Apgar score at 1 minute after birth were observed.

## 3. Statistical Analysis

IBM SPSS 24.0 software was used for data processing. The normally distributed data were expressed as mean ± standard deviation, the nonnormally distributed data were expressed as median and interquartile spacing, and qualitative data were expressed as composition ratio. We used the independent-samples *t* test, Mann–Whitney *U* test, and chi-square test to analyze the statistical differences. *P* < 0.05 was considered a statistically significant difference.

## 4. Results

### 4.1. Deliveries of Pregnant Women with Preeclampsia in Our Hospital during Four Years

From 2017 to 2020, a total of 87010 deliveries were made in our hospital, including 44601 deliveries from 2017 to 2018 and 42409 deliveries from 2019 to 2020. The delivery mode and delivery volume of pregnant women with preeclampsia are shown in Table 1. Statistical analysis results showed that the number of deliveries of preeclampsia from 2019 to 2020 increased significantly compared with the previous two years, and the rate of delivery of cesarean section due to vaginal trial delivery failure decreased compared with the previous two years.

### 4.2. Clinical Characteristics of Mothers and Newborns

The age distribution of patients with preeclampsia was 17∼45 years, the gestational week of delivery was 259∼291 days, and the number of pregnancies ranged from 1 to 6, and these in the control group were 18∼43 years, 259∼ 293 days, and 1∼8 times. In addition, there were 50 (39.37%) women in the study group and 32 (34.78%) women in the control group who had histories of childbirth. There were no differences in the demographic parameters of mothers and newborns between the two groups, as shown in Table 2 for details.

### 4.3. Vaginal Delivery Outcomes of the Two Groups

The vaginal delivery outcomes are compared between the two groups of preeclampsia women. We found that the duration of the first and second stages of labor was slightly shorter in the study group than in the control group, and the rates of episiotomy and postpartum hemorrhage volume within two hours were lower than those in the control group, but the duration of the third stage of labor, rate of forceps delivery, rate of cervical laceration, and placental abruption were not significantly different from those in the control group. See Table 3.

### 4.4. Comparison of the Causes of Postpartum Hemorrhage between the two Groups

A total of 39 patients in the two groups suffered from postpartum hemorrhage. The main causes of postpartum hemorrhage were uterine weakness, followed by placental factors and birth canal lacerations. No postpartum hemorrhage caused by coagulation dysfunction occurred. Statistical analysis showed that there was no difference in the causes of postpartum hemorrhage between the two groups. See Table 4.

### 4.5. Comparison of Hemostatic Methods between the Two Groups

The hemostatic measures of the two groups were mainly the combination of two pro-uterine contraction drugs, followed by a single pro-uterine contraction drug, and in a few cases, three contraction drugs or even uterine tamponade were used. Statistical analysis showed no difference in the methods of hemostasis between the two groups. The detailed results are shown in Table 5.

## 5. Discussion

In the context of rising cesarean section rate globally, according to the statistics of National Maternal and Child Health Care, the cesarean section rate in China increased from 28.80% to 36.70% from 2008 to 2018 [13], which seriously exceeded the alarm level of the cesarean delivery rate set by the World Health Organization [14]. At the same time, a series of serious complications caused by cesarean section, such as placenta previa, uterine incision pregnancy, placenta implantation, and uterine rupture, have seriously affected maternal safety and also impose heavy economic burden to the society. In recent years, vaginal delivery has been advocated worldwide to reduce the primary cesarean section rate [15], and in 2021, China's Health and Welfare Commission listed “reducing the incidence of vaginal delivery complications” as an improvement goal of medical quality and safety. As a common obstetric complication, preeclampsia affects a large number of women in China. It was not difficult to find that the incidence of simple preeclampsia in our hospital increased significantly in the past two years, and the number of pregnant women who directly chose cesarean section for various reasons also increased under the background of the continuous improvement of medical technology, which was contrary to the goal of improving medical quality and safety in China. Therefore, based on the safety of mother and baby, it is one of the key works of obstetricians to promote vaginal delivery of pregnant women with preeclampsia.

The introduction of the smart medical information system is one of the major initiatives to promote vaginal delivery in our hospital. In 2019, the hospital completed the interconnection of the outpatient electronic case system, remote fetal heart rate monitoring system, inpatient electronic case system, nursing system, testing system, and imaging system so that obstetricians could get a comprehensive and detailed understanding of patients' blood pressure fluctuations during pregnancy when receiving pregnant women with preeclampsia. Changes in blood test indicators, drug use, and fetal growth indicators are conducive to the development of detailed prenatal examination plans and reasonable delivery plans for patients and reduce misdiagnosis and missed diagnosis caused by incomplete and accurate patient history review. When the patients were sent to the delivery room to wait for delivery, the delivery room medical staff could also achieve good communication with outpatient doctors, ward doctors, and nurses through the medical information system, better observe the progress of labor, and give timely and accurate intervention measures according to the timely feedback of the central fetal heart rate monitor.

Intrapartum ultrasound is a technique of labor monitoring that has become popular in clinic in recent years. The monitoring includes fetal position, fetal head position, and fetal lie. Commonly used parameters include fetal head progression angle, midline angle, distance between fetal head and pubic symphysis, fetal head direction, and distance between fetal head and perineum. With the guidance of ultrasound imaging, we can quantify each parameter index to evaluate the progress of labor more accurately and to seize the right time to intervene in labor to avoid unnecessary vaginal-assisted labor and intermediate cesarean delivery. In the past two years, we have adopted the method of vaginal palpation combined with intrapartum ultrasound during labor to comprehensively evaluate the labor process. On the one hand, it avoided the misjudgment of labor process caused by inadequate clinical experience in obstetrics and inaccurate palpation of vagina, and on the other hand, it avoided the measurement error of parameters caused by incomplete ultrasound knowledge. Compared with the outcomes of the two groups, the duration of the first and second stages of labor in the study group was slightly shorter than that in the control group, and the rates of forceps delivery and perineal laceration were also lower than in the control group, while the rate of cesarean section and perineal lateral resection was significantly lower than that in the control group. The results of this study gave positive implications for the observation of labor progress of pregnant women with preeclampsia by vaginal palpation combined with intrapartum ultrasound.

While efforts are being made to promote vaginal delivery in preeclampsia, we need to be more proactive in preventing and reducing the delivery complications of preeclampsia. Pregnant women with preeclampsia are often accompanied by decreased proteinuria and plasma albumin levels and are prone to edema of the limbs and skin, as well as edema of the myometrium, which can lead to weak uterine contractions. Combined with the use of sedatives and antispasmodics during labor, the probability of postpartum hemorrhage due to weak uterine contractions will be higher. In this study, the main cause of bleeding in both groups was uterine contraction weakness. The median postpartum hemorrhage volume within two hours in the study group was 280 mL and the maximum bleeding volume was 1650 mL, while in the control group, they were respective 325 mL and 1500 mL. On the basis of the same uterine pathology in preeclamptic women, the age, gestational age, number of gravidities, parities and fetuses, causes of bleeding, and hemostatic measures in both two groups were basically the same, and the postpartum hemorrhage volume within two hours was less in the study group than in the control group. The possible reasons were considered as follows: (1) the extensive development of Doula delivery and labor analgesia services could relieve the tension of pregnant women with preeclampsia, avoid the drastic fluctuation of blood pressure during labor, and promote the changes in norepinephrine and other endocrine hormones to strengthen the contractile force of the uterus. (2) Warm life care, appropriate food, and fluid supplementation ensured adequate energy supply during labor, which not only reduced the failure of vaginal delivery due to insufficient maternal blood volume but also enhanced uterine contraction.

## 6. Summary

Under the environment of actively promoting vaginal delivery, reducing the rate of first cesarean section and the complication rate of vaginal delivery, actively promoting the construction of smart hospital, improving medical information system, ensuring convenient and adequate maternal and fetal monitoring equipment, and improving the quality of delivery services can not only effectively reduce the probability of failed vaginal trial of labor and perineal scoliosis in preeclamptic women but also effectively reduce the postpartum hemorrhage volume within two hours without increasing the use of hemostatic drugs. As obstetricians, we should strengthen our theoretical knowledge and skills in obstetrics, as well as our knowledge of psychology and ultrasound imaging, to deal with various emergencies that may occur during labor.

## Figures and Tables

**Table 1:** Preeclampsia deliveries in our hospital during four years.

	01/01/2017–31/12/2018	01/01/2019–31/12/2020	*P* value	Method
Total number of deliveries (cases)	44601	42409		
Preeclampsia deliveries (cases/rate)	261 (0.59%)	440 (1.04%)	＜0.001	Pearson's chi-square
Vaginal deliveries (cases/rate)	92 (35.25%)	127 (28.86%)	0.078	Pearson's chi-square
Cesarean delivery (cases/rate)	169 (64.75%)	313 (71.14%)	0.078	Pearson's chi-square
Births converted to cesarean section (cases/rate)	29 (17.16%)	33 (10.86%)	0.038	Pearson's chi-square

**Table 2:** Clinical characteristics of mothers and newborns of study population.

	Study group (*n* = 127)	Control group (*n* = 92)	*P* value	Method
Age (years)	28.65 ± 5.32	29.36 ± 5.62	0.340	Independent-samples t
Gestational age (days)	273.85 ± 7.68	275.47 ± 8.26	0.138	Independent-samples t
Gravidity (times)	2 (1, 3)	2 (1, 3)	0.598	Mann–Whitney
Parity (times)	1 (1, 2)	1 (1, 2)	0.520	Mann–Whitney
Neonatal weight (kg)	3.29 ± 0.42	3.29 ± 0.39	0.941	Independent-samples t
Apgar score at 1 minute after birth	10 (10, 10)	10 (10, 10)	0.091	Mann–Whitney

Data are presented as median (interquartile spacing) or mean ± standard deviation.

**Table 3:** Vaginal delivery outcomes of these study groups.

	Study group (*n* = 127)	Control group (*n* = 92)	*P* value	Method
Duration of the first stage of labor (minutes)	440 (245, 600)	480 (280, 750)	0.496	Mann–Whitney
Duration of the second stage of labor (minutes)	29 (16, 48)	31 (15, 60)	0.787	Mann–Whitney
Duration of the third stage of labor (minutes)	8 (5, 10)	8 (5, 10)	0.759	Mann–Whitney
Episiotomy (cases/rate)	39 (30.71%)	41 (44.57%)	0.042	Pearson's chi-square
Forceps delivery (cases/rate)	4 (3.15%)	4 (4.35%)	0.919	Continuity correction
Perineal laceration (cases/rate)	32 (25.20%)	24 (26.09%)	0.882	Pearson's chi-square
Cervical laceration (cases/rate)	7 (5.51%)	1 (1.09%)	0.174	Continuity correction
Postpartum hemorrhage volume within two hours (mL)	280 (200, 355)	325 (240, 433.75)	0.037	Mann–Whitney

Data are presented as median (interquartile spacing) or mean ± standard deviation.

**Table 4:** Comparison of causes of postpartum hemorrhage between the two study groups.

	Weak contractions (cases/rate)	Placental factors (cases/rate)	Birth canal laceration (cases/rate)
Study group (*n* = 15)	10 (66.67%)	3 (20.00%)	2 (13.33%)
Control group (*n* = 24)	18 (75.00%)	4 (16.67%)	2 (8.33%)
*P* value	1.000		
Method	Monte Carlo		

**Table 5:** Comparison of hemostatic methods between the two groups.

	One uterine contraction drug (cases/rate)	Two uterine contraction drugs (cases/rate)	Three uterine contraction drugs (cases/rate)	Uterine tamponade (cases/rate)
Study group	59 (46.46%)	62 (48.82%)	5 (3.94%)	1 (0.79%)
Control group	39 (42.39%)	48 (52.17%)	4 (4.35%)	1 (1.09%)
*P* value	0.932			
Method	Monte Carlo			

## Data Availability

The labeled dataset during this study is available from the corresponding author on reasonable request.
